# Research on Human Behavior Modeling of Sports Culture Communication in Industrial 4.0 Intelligent Management

**DOI:** 10.1155/2022/9818226

**Published:** 2022-03-01

**Authors:** Zhihui Li

**Affiliations:** Department of Physical Education, Lvliang University, Lv Liang, Shanxi 033000, China

## Abstract

With the advent of the information age, Internet technology and computer technology are gradually applied in various fields. Human daily life is inseparable from the help of information technology. The progress and development of the times are also changing our industrial environment. The Internet of things, artificial intelligence, and digital production have been widely used in the industrial field. We need to integrate the new intelligent management concept in the industrial 4.0 era into the modern industrial system and media communication. In the communication of sports culture, how to integrate the intelligent technology under the background of industry 4.0 and realize the spatiotemporal modeling and analysis of human behavior and behavior characteristics is the main content of our research. Firstly, this study briefly analyzes the development and historical process of industry 4.0 era and explores the impact of Internet of things and information technology on sports culture communication. This study analyzes the development process of Chinese sports culture communication and probes into the influence and significance of sports culture communication on human behavior. Under the background of industrial 4.0 management, a model of human temporal and spatial behavior change in sports culture communication is established. Human behavior trajectory is analyzed by data mining, human behavior recognition algorithm, behavior quantitative analysis method, and behavior feature model. The results show that under the background of industry 4.0 management, human behavior modeling can clearly describe the basic characteristics and behavior state in the process of sports culture communication and can predict and analyze the human behavior performance of such social activities and phenomena. Through data mining, data preprocessing, and behavior quantitative analysis, human behavior trajectory is studied. It has a positive impact on the behavior trend in human daily life. The main factor affecting behavior change is whether to receive sports culture news.

## 1. Introduction

With the continuous renewal of the development of industrialization, we divide the different periods of the industrial age into grades [1]. At present, it is roughly in the “4.0” era. The development mode, scale, and speed of industry are different in different industrial environments [2]. From the 18th century, Jenny textile machine changed the production efficiency and provided effective help for the liberation of human hands. Until Watt improved the steam engine, every industrial revolution was to make human work easier and easier [3, 4]. Traditional manual labor has been gradually replaced, and mechanical development and mechanical production have gradually become the main pillars of the industrial era. In the industrial 1.0 era, mechanical equipment manufacturing has become the main content of production mode in the whole period [5]. This defect is that the equipment covers an excessive area, and the production space can ensure the production demand through the increase of the number of machinery. Until the 20th century, the development of electric power has brought new opportunities to the fields of communication and automobile [6]. Human civilization began to move towards the industrial 2.0 era. The emergence of wired, wireless communication, chemical knowledge, and fuel vehicles has led to a sharp increase in the number of human labor in the industrial field. In the production environment, the division of labor is gradually clear, and the scale is further expanding. The new industrial level and equipment can bring more profits to enterprises [7]. Assembly line production is the main industrial process in this era. After World War II, the industrial 3.0 era began to enter people's lives. Machinery and equipment replace human labor and handicraft industry and become a substitute for assembly line enterprises [8]. The expansion of production scale no longer depends on the increase of the number of equipment but on the improvement of production methods and technical level. This era has further expanded the mode of mechanical equipment replacing human labor [9].

With the continuous development of human society and the progress of scientific and technological innovation and information technology, new opportunities have been brought to the industrial environment [10]. Scientific and technological innovation has led to great changes in human society. In order to accelerate the speed of scientific research achievements, many countries take the lead in setting up R&D centers such as scientific and technological manufacturing. Internet technology and information technology have also made great contributions to the advent of the industrial 4.0 era [11]. In project management, how to use big data technology to establish an intelligent management system is a key topic in each field. If managers cannot recognize the relationship between work needs and modern technology, they will not be able to adapt to the changes of the times. In the field of communication, the communication of sports culture in China has always been in a relatively weak link [12]. There is no deep-seated research on the impact of sports culture communication on human behavior.

This study is mainly divided into three structures: the first part briefly describes the development status of industry 4.0 model in various countries and analyzes the specific help provided by human behavior modeling research. The second part first explores the essence of sports culture communication in the industrial 4.0 environment and models the impact of sports culture communication on human behavior. Data mining and processing methods are used to analyze human behavior data, and modeling research is carried out from the spatial characteristics of human behavior. Finally, it analyzes the necessity of modeling human behavior characteristics in the communication of sports culture. The intelligent recommendation algorithm is used to actively realize the news prediction service of sports culture in the human behavior analysis model. The third part analyzes the research results of human behavior space modeling of sports culture communication under the environment of industry 4.0 and the research results of human behavior feature modeling.

## 2. Related Works

The core technology in the industrial 4.0 era is the field of Internet of things and information technology [13]. Communication technology and information development have played an important role in the industrial 4.0 era. Artificial intelligence can use electrified equipment and program calculation in Ronnie simulation to help analyze human behavior in the industry [14]. In the big data environment, processing huge information and complex data sets also need to use big data for mining and processing. Big data technology can provide effective and accurate data for industrial 4.0 intelligent management, intelligent transportation, intelligent production, and other modes and help industrial development move forward steadily [15]. In Internet computing, cloud computing can provide information and software resources for management devices and analysis devices. When big data collects and analyzes information, heterogeneous distribution, measurement, and other functions can be realized by using cloud computing [16]. The above are the main technologies ahead of the industrial 4.0 era. They provide technical support for the progress of the industrial era. The analysis, detection, and modeling of human behavior are often complex, but the efficient management function can be realized by using various modern technologies in the industrial 4.0 environment. We analyze the development status of countries in the industrial 4.0 era as follows [17]:

With the implementation of the industrial 4.0 era, Germany has made new changes in talent training mode. The dual system can improve the selection of talent training objectives, structural system, and professional ability training [18]. It puts forward new challenges for the types of talent training. With the gradual reduction of the matching between postwork and actual ability, enterprises pay more and more attention to the ability level of recruiters. The optimization of talent training program in vocational education schools is also a major problem to be solved. Facing these challenges, German vocational schools put forward the dual system training management model. The industrial 4.0 environment complies with the development of the times, expands the direction of professional development, and transports professional talents for the country [19].

The development of information technology and modern industry in the United States is relatively advanced, and they have always been in a leading position in the process of industrial reform [20, 21]. With the continuous application of modern equipment, the manufacturing industry is also in urgent need of improving its own technology. Under the environment of industry 4.0, there is a higher demand for equipment manufacturing and equipment manufacturing industry. Intelligent reform has become the main direction of industrial 4.0 mode. The intelligent management of robot equipment in industrial operation has also become the main topic. They applied the sensor technology of Internet of things in the industrial 4.0 era to the transformation of industrial robots and realized the intelligent development to a certain extent [22].

The apprenticeship reform system in Italy has changed with the advent of the industrial 4.0 era [23, 24]. When the apprenticeship reform becomes the focus again in the world, Italy's national and regional management system puts forward new policies for the apprenticeship reform. In terms of system management, innovative measures have been taken in the application of industrial 4.0 intelligent management, curriculum development, and quality inspection. Under the industrial 4.0 environment, different types of apprenticeship systems can be positioned differently, realizing the effect of system optimization.

Taking Hong Kong and Macao as examples, China has transformed the manufacturing industry under the background of industry 4.0 to intelligent development [25]. Enterprises in the manufacturing industry are prone to many internal problems in the process of transformation. In this case, intelligent management in the era of industry 4.0 can help Hong Kong and Macao quickly change to the intelligent manufacturing industry. This study puts forward effective countermeasures and suggestions for its development path and solving problems. Based on industry 4.0 intelligent management environment, this study analyzes the human behavior modeling of sports culture communication.

## 3. Research on Human Spatiotemporal Behavior Modeling and Behavior Characteristics of Sports Culture Communication Based on Industrial 4.0 Intelligent Management

### 3.1. Intelligent Management of Sports Culture Based on Mobile Network

The main features of the industrial 4.0 era include interconnection. Connecting all things has always been the theme of the industrial 4.0 era. The universality of the connection scope can closely gather equipment, manufacturers, enterprises, communication institutions, users, and other objects together. In order to comply with the development trend of the Internet of things, the sensor equipment, intelligent management system, embedded equipment, mobile communication equipment, and intelligent communication equipment of the Internet of things constitute an intelligent network model. The production process of the factory can also be highly intelligent. Intelligent factories can be controlled by the Internet of things. That is, the production process is completely integrated by computer. The real-time production monitoring program knows what new materials and processes are needed to ensure the smooth progress of the production process. This is not a simple problem of production automation but the realization of intelligent control. If the system detects a sudden failure in the production process, the machine will automatically suspend operation and repair itself, rather than continue to operate and continuously produce defective products. Through information technology, the most effective utilization of energy can be ensured, which are the characteristics of intelligent chemical plants in the future.

It can integrate digital development with the physical world and connect with each other, so as to ensure that human society can live more conveniently. Every industrial revolution can help human progress. We analyze the process of industrial development in time and space, as shown in Figure 1.

As can be seen from Figure 1, industry 4.0 is a new era and its development time is expected to be long. With the advent of the new era, human behavior has gradually changed in diversity. We focus on sports culture communication.

Sports is a complex object in the development of social culture. It can combine the body and spirit as the basis of daily activities. With the continuous improvement of human growth and development, the mastery of sports and skills can ensure the healthy growth of physical quality. In order to achieve the all-round development of quality education, improve the physical quality of the whole people, and improve the way of life, we need to pay attention to the dissemination of sports culture. Although China's economic development is relatively rapid, it has not brought significant results to China's sports communication. We compare the gap between Chinese and foreign media in sports culture communication, as shown in Figure 2.

As can be seen from Figure 2, with the increase of years, China's attention to sports culture communication has gradually increased. But in 2010, it still cannot be compared with western countries. With the advent of the industrial 4.0 era, intelligent devices and the Internet have brought diversified development to human behavior. From the perspective of media communication mode, sports communication has an indispensable relationship with the development of Internet data. We make statistics on the data of Internet users and show the process of users obtaining sports and cultural news by means of mobile communication, wired Internet access, wireless Internet access, and virtual communication, as shown in Figure 3.

The continuous increase of survey behavior data is shown in Figure 3. From the beginning of mobile communication business, it has been transforming to wired Internet and wireless Internet. With the change of industry 4.0 era, virtual Internet also gradually exists in people's daily life. Therefore, the factors affecting human behavior by the dissemination of sports culture in the industrial 4.0 era are significant. We conduct modeling research on human behavior. Firstly, we analyze the range changes of individuals in time and space:

(1) $$\begin{array}{c} B≔\left\{\left(s_{i},t_{i},c_{i}\right)|i=0,1,2,...\right\}. \end{array}$$

In the formula, *B* represents the time-space behavior sequence, and (*s*_*i*_, *t*_*i*_, *c*_*i*_) represents the element set. The range of each element in the collection is expressed as follows:

(2) $$\begin{array}{c} b=\left(s,t,c\right)\in B,\;s\in D^{\left|s\right|}. \end{array}$$

We analyze that the spatial diffusion of human behavior change trajectory is decreasing. In the sample data, the data of users who are concerned about the dissemination of sports culture actively hiding information are analyzed. It can be found that the spatial change of human behavior is an exponential distribution. The mathematical formula can be expressed as follows:

(3) $$\begin{array}{c} p\left(\lambda \right)∼{\left(\lambda +\lambda_{0}\right)}^{-b}\cdot e^{\left(\lambda /k\right)}. \end{array}$$

The distribution of exponential function is between 0 and 2. Different cultural news takes different values. In the analysis of human spatiotemporal behavior, we need to observe from multiple angles. The spatiotemporal movement variation of each individual can be defined as follows:

(4) $$\begin{array}{c} R_{g}^{2}=\frac{1}{n}\sum_{k=1}^{n}{\left(r_{k}-r\right)}^{2}. \end{array}$$

In the formula, *R*_*g*_^2^ represents the characteristics of human behavior. We calculate the function law satisfied by the distribution of human behavior by using the transfer structure. The formula is as follows:

(5) $$\begin{array}{c} p\left(\lambda \right)=\int_{0}^{\infty }P\left(\lambda |R_{g}\right)P\left(R_{g}\right)\text{d}R_{g}. \end{array}$$

According to the above formula, the spatiotemporal pattern of human behavior can be determined. The law is calculated from the track data of the impact of sports culture communication on human behavior in the industrial 4.0 environment. Behavior pattern modeling can conform to the general process of human cognition. From the observed objects, it is found that many users have common characteristics. At present, more and more countries begin to pay attention to human behavior research. From the early stage of industry to 4.0, there are more and more technical means to study the human behavior model. We consulted relevant literature and analyzed the content release trend of human behavior modeling research over the years, as shown in Figure 4.

It can be seen from Figure 4 that the development of the industrial age has a great impact on human behavior modeling. Since 2015, the number of human behavior modeling literature published in China has increased significantly. However, compared with the foreign release, it is still in a weak position. In order to further explore the impact of sports culture communication on human behavior, we also need to study from the analysis of behavior characteristics.

### 3.2. Research on Sports Culture Communication Based on Industry 4.0 Intelligent Management in Human Behavior Feature Modeling

In China's sports, table tennis and volleyball have always been the proud contents of the people. In the process of talking about sports news, the dissemination of cultural knowledge is realized. As China continues to win the Olympic Games, people all over the country begin to discuss sports news. People's attention to sports events is also the main manifestation of their attention to sports culture. Government communication and people's communication are the main channels. However, the way of sports culture communication should focus on itself. This communication effect is not only related to the development of national influence but also has an important impact on the performance of people's daily life and behavior.

Under the background of industry 4.0, the information communication model based on human behavior characteristics can more accurately describe the effect and process of sports communication. The main advantage is that it can choose the response after receiving information according to the set of human behaviors, including evaluation, forwarding, no response, and so on. Modeling human behavior can simulate the effect of data transfer in a variety of states. In sports culture communication, modeling based on human behavior characteristics can monitor the process of culture communication, which is a process from individual to collective modeling. It can take into account the personalized behavior judgment of users, so as to realize accurate information push and other functions. With the gradual application of industry 4.0 management in Internet information dissemination, network data and human behavior data indices increase. In order to facilitate accurate push of everyone's behavior data, we need to conduct personalized behavior feature modeling. Before behavior feature analysis and modeling, we compare the data acquisition speed of intelligent management system in industrial 4.0 environment with that of traditional data mining system, as shown in Figure 5.

As can be seen from Figure 5, with the increase of massive information in big data environment, the acquisition speed of traditional data mining system tends to decrease. The intelligent management data system in industrial 4.0 environment can effectively judge accurate data and useless data and realize the function of rapid acquisition. In the estimation of human behavior characteristics, we use mathematical formula as follows:

(6) $$\begin{array}{c} \text{Interest}\left(w\right)=f\left({\text{Interest}}_{\text{Activit}}\left(w\right),{\text{Interest}}_{\text{Freq}}\left(w\right),{\cdot \text{Interest}}_{\text{Time}}\left(w\right)\right). \end{array}$$

Interest_Activit_ is the actual action of human behavior, and Interest_Freq_(*w*) represents the number of information access. In order to study the number of human information browsing actions, we define the calculation function as follows:

(7) $$\begin{array}{c} \left({\text{Interest}}_{\text{Activit}}\left(w\right)=f\left(\text{Sava}\left(w\right)\right.,\text{Keep}\left(w\right),\text{print}\left(w\right),\text{Copy}\left(w\right)\right). \end{array}$$

Among them, they respectively represent the times of saving, collecting, and printing sports culture web pages and forwarding of information content. The browsing action can be represented by a binary function. The specific formula is as follows:

(8) $$\begin{array}{c} {\text{Interest}}_{\text{Activit}}\left(w\right)=\left\{0,\text{Sava}\left(w\right),\text{Keep}\left(w\right),\text{print}\left(w\right),\text{Copy}\left(w\right)\right\}, \end{array}$$

(9) $$\begin{array}{c} {\text{Interest}}_{\text{Activit}}\left(w\right)=\left\{1,\text{Sava}\left(\varpi \right),\text{Keep}\left(\varpi \right),\text{print}\left(\varpi \right),\text{Copy}\left(\varpi \right)\right\}. \end{array}$$

Investigation shows that most users rarely save and collect web pages when browsing sports culture news. Therefore, we cannot fully obtain the overall behavioral characteristics of human beings by using behavioral interest analysis. We need to calculate the number of visits and residence time respectively, so as to realize the feature modeling of human behavior. The number of behavior-based stops can be expressed by the following function:

(10) $$\begin{array}{c} {\text{Stop}}_{\text{Freq}\left(w\right)}=\frac{\text{Freq}\left(w\right)}{\underset{E\in W}{\max}\left(\text{Freq}\left(w\right)\right)}. \end{array}$$

Among them, *w* represents the number of news visits by users in a certain period of time. With the increase of time, the number of behaviors is also accumulating. We update the number of visits in a cycle in the formula in proportion. In mathematical calculation, it can be calculated according to the following equation:

(11) $$\begin{array}{c} p=\frac{\left(|{\text{Freq}}_{\text{new}}\left(w\right)-{\text{Freq}}_{\text{old}}\left(w\right)|\right)}{{\text{Freq}}_{\text{old}}\left(w\right)}, \end{array}$$

(12) $$\begin{array}{c} \text{Freq}\left(w\right)=\left({\text{Freq}}_{\text{new}}\left(w\right)+{\text{Freq}}_{\text{old}}\left(w\right)\right). \end{array}$$

When the coefficient *p* is less than 0, it represents human behavior, and the number of visits of users in the cycle does not change significantly. This study defines the browsing speed of each page of sports culture communication page as follows:

(13) $$\begin{array}{c} \text{Speed}\left(w\right)=\frac{\text{Size}\left(w\right)}{\text{Time}\left(w\right)}, \end{array}$$

where size(*w*) represents the storage size of the propagation interface and time(*w*) represents the time coefficient. Finally, the data delay in the management interface is calculated as follows:

(14) $$\begin{array}{c} \text{Time}\left(w_{i}\right)=T\left(w_{j}\right)-T\left(w_{i}\right). \end{array}$$

Next, the coefficient of influence on human behavior characteristics in the process of sports culture communication is calculated as follows:

(15) $$\begin{array}{c} R=\frac{{\text{Interet}}_{\left(w\right)}}{\left(\text{Speed}\left(w\right)/\max_{E\in W}\right)}. \end{array}$$

According to the above formula, we can model the characteristics of human behavior and explore the impact of sports culture communication on human behavior under the management of industry 4.0. In the sports culture communication interface, we use the nonlinear normalization method to process the sample data. Compared with the traditional processing method, we compare the error coefficient, as shown in Figure 6.

As can be seen from Figure 6, the error coefficient of the traditional processing mode begins to increase with the increase of human behavior data. The data processed by nonlinear normalization can maintain basic accuracy.

## 4. Modeling of Human Spatiotemporal Behavior and Analysis of Behavior Characteristics Based on Sports Culture Communication in Industrial 4.0 Intelligent Management

### 4.1. Analysis of Research Results of Human Spatiotemporal Behavior Modeling of Sports Culture Communication Using Mobile Network in Industrial 4.0 Intelligent Management

In the industrial 4.0 environment, the intelligent management mode can liberate human labor and realize behavior interaction and industrial production on the basis of human wisdom. This model can optimize the traditional communication mechanism into intelligent communication mechanism in the field of communication and provides the core technology in human behavior analysis and modeling. Dealing with the invisible factors in the Internet era can change the performance and accuracy of human behavior model from uncontrollable to controllable under the premise of massive data. Firstly, we analyze the accuracy change of data in the process of human behavior modeling in the industrial 4.0 environment, as shown in Figure 7.

It can be seen from Figure 7 that the traditional human behavior model cannot guarantee the accuracy of data in the modeling process based on the massive data in the Internet age. The human behavior model in the industrial 4.0 environment can ensure the processing speed and control the accuracy above the standard range. In the mobile network environment, sports culture communication can be guaranteed. We build a human behavior model on mobile users. In the above calculation process, it is found that there are strong temporal and spatial characteristics and scene factors in the behavior participation characteristics of mobile networks. These scene factors are easily affected by many aspects. For example, the response of surrounding people to cultural news can indirectly affect individual behavior changes. We use objective quantitative method to map human behavior participation modeling. The response behavior influence coefficient of people in three states to sports cultural news is analyzed, as shown in Figure 8.

As can be seen from Figure 8, the influence coefficient of the crowd who obtains sports news is relatively stable, and the influence coefficient of the crowd who indirectly obtains news information is relatively severe. The influence coefficient of people who do not get sports news is low. The above trends of human behavior can well explain that the impact of sports culture communication on behavior characteristics is significant.

### 4.2. Analysis of Research Results of Sports Culture Communication of Industry 4.0 Intelligent Management in Human Behavior Feature Modeling

In an intelligent video surveillance system, the accuracy of background model has an important impact on the subsequent judgment of foreground detection, classification, tracking, and behavior understanding analysis. In other words, it largely determines the performance of the whole video surveillance system. Complex scenes greatly increase the impact on the accuracy of model monitoring. The human behavior modeling process faces complex scenes in the industrial 4.0 environment, which will be affected and changed by many aspects of the outside world. Human beings may have a variety of behavior characteristics under the specified time and space sequence, or there may be no characteristic changes. Therefore, in the detection process, we need to locate and analyze from the initial cause to the behavior space. The calculation is based on the modeling of human behavior characteristics, including the judgment of the change of user interest. At different times, people staying in the same news can have different effects on the calculation results. With the increase of human behavior data, we need to study feedback efficiency in the model. The feedback speed of human behavior characteristic data before and after industrial 4.0 intelligent management is mainly compared, as shown in Figure 9.

As can be seen from Figure 9, the traditional management mode cannot meet the needs of efficient feedback in the dynamic change characteristics of data. The intelligent management mode in the industrial 4.0 environment can help the analysis model of human behavior characteristics to ensure the feedback efficiency. In the verification process of this study, the main flow of data feature processing is shown in Figure 10.

As can be seen from Figure 10, firstly, in data mining, we capture the main content of sports culture on an Internet platform. Secondly, the obtained data are preprocessed to facilitate the analysis of key features. The basic structure of the Internet is extracted, and the form of active behavior is taken as the general category of data statistics. Finally, the data distribution principle is used for visual analysis, and the characteristic changes of human behavior are verified by hypothesis theory. In the final experimental results, we found that there are positive and negative trends in the impact of sports culture communication on human behavior under the industrial 4.0 Internet mode.

## 5. Conclusion

This study proposes to model the human behavior of sports culture communication in the industrial 4.0 intelligent management environment. Firstly, it analyzes the development process of industrial 4.0 environment and the current situation and difficulties of sports culture communication in China. Through data mining, data preprocessing, and behavior quantitative analysis, human behavior trajectory is studied. Under the condition of sports culture communication, the temporal and spatial changes of human behavior are modeled. The influencing factors of human behavior are divided into multiple models to calculate the data distribution of the temporal and spatial characteristics of individual behavior. Based on individual data set, it is transformed into the statistical analysis of group behavior. Finally, according to the track of human behavior and historical traces, the specific factors affecting behavior changes are analyzed. Search modeling is used to explore the characteristic changes of human behavior. The results show that in the industrial 4.0 environment, the communication mechanism and industrial process have changed by leaps and bounds. The results of this study have a positive impact on the behavior trend in human daily life. The main factor affecting behavior change is whether to receive sports culture news. It promotes the process of traditional culture communication and especially helps the communication of sports culture form a good cycle. In order to explore the process of the influence of sports culture news on human behavior. However, this study does not carry out simulation verification analysis on the model data, and further elaboration is needed in future research.

## Figures and Tables

**Figure 1:** Industrial development process.

**Figure 2:** The gap between Chinese and foreign media in sports culture communication.

**Figure 3:** The process of obtaining sports culture news in various ways.

**Figure 4:** The content release trend of human behavior modeling research over the years.

**Figure 5:** Comparison of data acquisition speed between the system and traditional data mining system.

**Figure 6:** Comparison of error coefficient between traditional processing method and nonlinear normalization processing method.

**Figure 7:** Accuracy changes of human behavior modeling data in industrial 4.0 environment and traditional models.

**Figure 8:** Influence coefficient of response behavior of people in three states to sports cultural news.

**Figure 9:** Feedback speed of human behavior characteristic data before and after industrial 4.0 intelligent management.

**Figure 10:** Main flow of data feature processing.

## Data Availability

The data used to support the findings of this study are available from the corresponding author upon request.
